The article "Sports Energy Consumption Evaluation Based on Improved Adaptive Weighted Data Fusion Energy-Saving Algorithm" was published in 2022. Journal: Comput Intell Neurosci.

# Sports Energy Consumption Evaluation Based on Improved Adaptive Weighted Data Fusion Energy-Saving Algorithm

**DOI:** 10.1155/2022/7261193

**Published:** 2022-04-22

**Authors:** Ling Han, Yanping Jiang

**Affiliations:** Xi'an Medical University, Xi'an City, Shaanxi Province 710021, China

## Abstract

The purpose of this study is to use a portable cardiopulmonary function tester to measure the effect of sports smart bracelets and smartphone application software in monitoring the energy consumption of different types of physical activities, and to select several popular sports software in daily life for research. The tester is an accurate reference value. It compares the energy consumption monitoring effect and error percentage of several software in periodic exercise and discusses the relationship between the measured value and reference value of several software, so as to provide a scientific basis for exercise for the majority of athletes. The selection of software provides a reference and chooses a more suitable movement method according to its own actual situation to achieve the most objective and effective periodic movement. In this study, the CMA (constant modulus algorithm) is introduced into the decision feedback equalizer, and the CMA-DFE (decision feedback equalization) algorithm is formed. Since the CMA algorithm adopts a fixed step size, there is no way to solve the contradiction between the convergence speed and the steady-state residual error, so a constant modulus algorithm with a variable step size is proposed. The algorithm increases the step size in its initial stage to increase the convergence speed and reduces the step size after the algorithm converges to reduce the steady-state residual error. This study replaces the traditional CMA algorithm with the constant modulus algorithm with a variable step size. In this section, two basic algorithms for calculating the adaptive weighting factor are first proposed. Due to its limitations, a modified adaptive weighting factor is proposed. During normal running, the Huawei Band relatively accurately monitors the number of steps and energy consumption, and the motion software of the motion software relatively accurately monitors the distance. The monitoring of distance and energy consumption is relatively accurate in the Codoon sports software; in jogging, the Huawei Band is relatively accurate in monitoring the number of steps; the LeDong sports software is relatively accurate in monitoring distance; and the Codoon sports software in the energy consumption is relatively accurate.

## 1. Introduction

In the scientific field of sports and fitness, scientific researchers can use acceleration sensors and other instruments such as accelerometers to effectively extract and analyze fitness data, and can obtain ideal results [1]. These devices can not only provide information about physical activity, the number of steps, exercise distance, duration, energy consumption, and other information are also quite accurate after being verified by multiple methods and multiple researchers [2]. However, these smart devices are used in scientific research after all. Due to the high price of devices such as accelerometers and complicated data collation, they need to be operated by relevant professionals. Therefore, they cannot be used in mass sports and cannot be used for mass fitness. It is not suitable for monitoring the amount of physical activity of the public during exercise. There are many kinds of human body movements, but most people still use periodic walking and running movements. For this reason, how to measure the energy consumption of the human body during the movement process more objectively, reliably, conveniently, and accurately needs to be discussed. The method of human energy consumption must be suitable for long-term use by most people, and the measurement must be simple, inexpensive, and easy to carry out other activities that do not affect the human body. With the continuous development of science and technology, smart bracelets and smartphones are gradually accepted by the public because they are easy to carry, can obtain intuitive data, and can analyze the amount of exercise through the measured energy consumption value [3]. Therefore, it is necessary to study the effects of portable smart devices such as smart bracelets and smartphones in measuring the energy consumption of different walking and running methods, so as to provide a reference for public fitness.

Physical fitness can be comprehensively improved through physical activity. It can accelerate blood circulation in the brain, promote metabolism, enhance cardiopulmonary function, significantly reduce weight, and play a positive role in mental health [4]. In recent years, with the development of the internet and the emergence of smartphones, various mobile phone sports software can monitor the daily physical activity of people [5]. Compared with the energy consumption instruments in the laboratory, smartphones are more friendly to people and will not cause economic damage to the wearer. If the built-in acceleration sensor in smartphones can effectively evaluate sports, it is bound to be able to guide the public to scientifically do sports. Some foreign researchers have conducted quantitative research on sports such as walking, jogging, moderate-speed running, cycling, and stair climbing through smartphone sports software [6]. For this reason, it is necessary to use the built-in accelerometer of smartphones to establish an effective prediction equation for sports, whether from the perspective of the accuracy of energy consumption assessment by built-in accelerometers in smartphones or the gap between related research at home and abroad. Due to the particularity of sports, sports software may not be suitable for sports monitoring, and the energy consumption algorithm of smartphone sports software on the market is a commercial secret, and researchers have no way of knowing [7]. Therefore, this study will discuss the processing process of the raw acceleration signal of the fitness skipping rope by the built-in acceleration sensor of the smartphone, establish a processing method suitable for the raw acceleration signal of sports, then enrich the internal algorithm of the smartphone, and provide a theoretical basis for scientific fitness.

The adaptive equalizer performs “inverse filtering” on the received signal sequence to offset the multipath effect intersymbol interference, but it has a premise that the transmitter needs to send the training sequence uninterrupted. However, the blind equalizer does not require the transmitter to continuously send the training sequence to compensate for channel distortion. It does not need to externally provide the expected response, and it can generate and restore the input signal sequence that is expected to be restored. The output of the filter is best approximated under some criterion (MMSE criterion). This study extracts the characteristic parameters of the acceleration signal, describes the feature extraction process of the acceleration signal collected by the experiment, introduces the relevant theories used in the process of the acceleration signal processing, extracts the characteristic parameters of the signal, and performs the characteristic parameters. The difference is a significant sex test. During normal running, the Huawei Band relatively accurately monitors the number of steps and energy consumption, and the motion software of the motion software relatively accurately monitors the distance. The monitoring of distance and energy consumption is relatively accurate in the Codoon sports software; in jogging, the Huawei Band is relatively accurate in monitoring the number of steps; the LeDong sports software is relatively accurate in monitoring distance; and the Codoon sports software in the energy consumption is relatively accurate. These five types of exercise software are not very effective in monitoring energy consumption, and there are large errors in fitness exercise. Compared with other exercise methods, the measurement results of each software have smaller errors when jogging. Compared with other software, the error rate of the Codoon exercise software and Huawei Bracelet is lower.

## 2. Related Work

Data-driven methods can be classified according to the scenario [8]. These methods are all to save energy and reduce the amount of data sent to the sink node, but their principles are different. Data reduction is mainly aimed at unnecessary sampling problems, while energy-efficient data acquisition mechanisms are mainly aimed at energy saving in the perception subsystem. In-network data processing performs data processing on the current node to reduce the amount of data transmitted. In practical applications, this method will be very different due to different scenarios [9].

Regarding the energy consumption of wireless sensor network nodes, in general, it is considered that the energy of communication is much higher than the energy consumption of sampling and calculation. Therefore, in general research, the energy consumption of sampling is negligible. But there are some scenarios where this assumption does not apply. In fact, for a large number of sensors, the energy consumption of sampling is also very large, even exceeding the energy consumption of communication [10, 11].

Adaptive sampling technology studies the correlation between data and reduces the number of samples [12]. For example, the changes in the data in the time series are relatively gentle. Time correlation can be used to reduce the number of samples. Similarly, by using spatial correlation, the sampling of adjacent nodes can be uniformly organized. Therefore, temporal and spatial correlations can be combined to reduce the number of samples.

In recent years, for sensor applications with high sampling energy consumption, methods for controlling the sampling frequency of nodes have emerged [13]. These methods focus on how to control the sampling frequency, that is, “selective sampling” or “adaptive sampling.” Different from data compression and communication compression technology, adaptive sampling technology uses the spatial and temporal correlation between data to dynamically adjust the sampling rate, which is a method to reduce the amount of sampling.

Heart rate during exercise is closely related to the volume and intensity of exercise training. The heart rate during exercise is mostly used to observe the exercise intensity of athletes. It can be read at any time through the telemetry heart rate monitor or by measuring the heart rate immediately after the exercise. The method is to measure the number of pulses within 10 s or 30 s to calculate the unit time [14]. This method is mostly used in daily exercise and is not limited by sports equipment. Within a certain range, the greater the exercise intensity, the higher the exercise heart rate, and the two are linearly related, especially when the body reaches a stable state, the heart rate and exercise intensity are positively correlated, and when the training load is large, the athlete will experience fatigue, manifested as basal heart rate (i.e., resting heart rate) that rises faster [15]. All these theories provide a theoretical basis for indirectly measuring the body's energy consumption and controlling the intensity of the aerobic exercise by using exercise heart rate. Professional sports coaches will also use heart rate monitoring to determine the training intensity and amount of exercise of athletes, and adjust exercise training plans according to the physiological response of athletes to improve the effect of exercise training [16]. College students are the main force of colleges and universities. They have the characteristics of a large group base and obvious differences between individuals and majors, and physical exercise is limited by venue and time, and lack of professional sports knowledge. Therefore, in the process of physical exercise, there are often differences in exercise methods and load arrangements.

Calories (or joules) are a common unit of energy consumption, and energy intake is usually calculated in calories (or joules) [17]. Therefore, when evaluating energy consumption, the oxygen uptake measured by gas metabolism is usually converted into calories, which means that under normal circumstances, oxygen uptake can be directly converted to calories (or joules) per minute, and studies have shown that per liter of oxygen can release 4.7 kcal of calories from fat, so calories (or joules) per minute are one of the most intuitive representations of energy expenditure [18].

## 3. Methods

### 3.1. Blind Equalization Algorithm Based on Decision Feedback

The linear equalizer has a simple structure and relatively stable performance. However, when the channel has a zero point close to the unit circle, that is, when the channel frequency selective fading is severe, the filter will form a large gain at the corresponding position in order to compensate for the channel distortion, thereby greatly increasing the additional noise in the received signal. The decision feedback equalizer can effectively eliminate the intersymbol interference without introducing noise gain because of the nonlinear characteristics of the feedback filter.

For the receiver using the adaptive algorithm (LMS), it is usually necessary to transmit a training sequence for equalization. However, in the system of high-speed wireless digital communication, the existence of a multipath effect makes the channel distorted. Even if adaptive equalization is used in this case, the success of extracting the training sequence is determined by the normal operation of the carrier recovery loop [19–21]. Therefore, if the carrier recovery is suddenly interrupted, the training sequence cannot be successfully extracted, and the equalization will fail [22]. The block diagram of the CMA-DFE structure is shown in Figure 1. In the figure, *a*(*k*) is the zero-mean IID transmit signal, *H*(*z*) is the channel impulse response, *v*(*k*) is the noise gain, and *x*(*k*) is the input sequence of the feedforward equalizer, which is defined as follows:

(1) $$\begin{array}{c} x\left(k\right)=\sum a\left(k-i\right)h_{i}\left(k\right)-v\left(k+1\right). \end{array}$$

It is assumed that the tap length of the feedforward transversal filter is *N*_1_, and the tap length of the feedback transversal filter is *N*_2_. The final output sequence *z*(*k*) of the decision feedback equalizer is the difference between the output sequence *y*_*f*_ (*k*) of the feedforward transversal filter and the output sequence of the feedback transversal filter:

(2) $$\begin{array}{c} z\left(k\right)=\left|y_{b}\left(k\right)-y_{f}\left(k\right)\right|=w_{f}\left(k\right)x^{T}\left(k-1\right)-w_{b}\left(k\right)a^{T}\left(k+1\right). \end{array}$$

The CMA algorithm is now used to update the weights of the feedforward equalizer and the feedback equalizer. The cost function of the CMA algorithm is as follows:

(3) $$\begin{array}{c} J_{c}\left(k\right)=E\left[e\left(k-1\right)\cdot e\left(k\right)\right]. \end{array}$$

The error function is defined as follows:

(4) $$\begin{array}{c} e\left(k\right)=\left|z\left(k\right)\cdot z\left(k+1\right)-R^{2}\right|. \end{array}$$

Then, the iterative formulas of the weight coefficients of the feedforward equalizer and the feedback equalizer are as follows:

(5) $$\begin{array}{c} w_{f}\left(k+1\right)=w_{f}\left(k-1\right)+u_{f}e\left(k-1\right)x\left(k-1\right),\\ w_{b}\left(k+1\right)=w_{b}\left(k-1\right)+\left|u_{b}e\left(k-1\right)a\left(k-1\right)\right|. \end{array}$$

### 3.2. Improved CMA-DFE Algorithm

It is assumed that the optimal weight vector of the tap weight coefficient of the equalizer is as follows:

(6) $$\begin{array}{c} W^{\prime }\left(k\right)=v\left(k\right)h_{i}\left(k+1\right)-z\left(k\right)e\left(k+1\right). \end{array}$$

Then, there are the following:

(7) $$\begin{array}{c} x^{\prime }\left(k\right)=W^{\prime }\left(k\right)Y\left(k-1\right)-\delta \left(k\right)e\left(k\right), \end{array}$$

where *δ*(*k*) is Gaussian white noise.

When the CMA algorithm converges, that is, the process in which the tap weight vector *W*(*k*) of the equalizer gradually approaches the optimal weight vector, the residual error will gradually decrease with the approximation process of the equalizer tap weight vector. Thinking of the step size factor of the CMA algorithm, in order to solve the contradiction caused by the fixed step size of the algorithm, it is necessary to use a large step size factor in the early stage of the algorithm to speed up the convergence speed. When the algorithm tends to converge, the algorithm adopts a small step factor to make the steady-state residual error small. This means that the change in the step factor is a decreasing process. The change process of the residual error in the CMA algorithm is exactly a decreasing process. The variation of the step factor can thus be controlled using the residual error.

However, if the residual error is directly used to control the step size change, there will be some defects. This is because interfering signals will have an impact on the residual error as the CMA algorithm gradually converges. Especially after the CMA algorithm tends to converge, if a strong interference signal suddenly appears, the residual error will suddenly increase, and the steady-state residual error will also increase, which may cause the algorithm to diverge. Therefore, directly using the residual error to control the step size factor cannot ensure the improvement of the performance of the CMA algorithm.

Directly using the residual error to control the step size change cannot effectively improve the performance of the CMA algorithm. However, it cannot be said that the residual error cannot be used to control the change in the step size, and it is only necessary to perform a certain mathematical transformation on the residual error to achieve the purpose.

Therefore, the variable step size algorithm based on the MSE transform can effectively solve the problem caused by the use of a fixed step size factor, that is, the contradiction between the convergence speed and the steady-state residual error. Therefore, the variable step size algorithm based on the MSE transform can be used to adjust the weight vector coefficients of the feedforward equalizer and the feedback equalizer of the decision feedback equalizer to form an improved algorithm. The algorithm structure diagram is shown in Figure 2.

There is a decider in the decision feedback equalizer. Hard decision judgment is usually used, that is, the output value of a symbol is 0 or 1 after the judgment is made. This kind of judgment will lose some interference characteristics of the channel, such as amplitude-frequency characteristics and phase-frequency characteristics, resulting in misjudgment. The decision feedback equalizer needs to make a decision on the received signal and use the decision signal as the input of the feedback equalizer. When an error occurs in the decision of a certain symbol by the decider, the wrong symbol will be propagated to the entire tapped delay line of the feedback equalizer. Not only that, it may affect consecutive symbol-incorrect decisions.

The core idea of the adaptive weighting algorithm is based on the adaptive weighting factor, and the output signal of the decider is judged according to the adaptive weighting factor. The adaptive weighting factor is a computable quantity between 0 and 1 that measures the accuracy of the decision output. The value of the adaptive weighting factor is usually realized by calculating the distance between the output of the feedforward equalizer and the constellation point.

The decision of the decider is only the adaptive weighted sum of hard decisions and undecided. Although it can effectively reduce the misjudgment phenomenon of the decision feedback equalizer, it will still cause a large degree of misjudgment. Therefore, a modified adaptive weighting algorithm is proposed on this basis. According to the analysis of the decision feedback equalizer, the outputs of the feedforward filter and the feedback filter can be expressed as follows:

(8) $$\begin{array}{c} x\left(n\right)=\overset{L_{f}}{\underset{i=0}{\prod }}\left[f_{i}\left(n-2\right)r\left(n-1\right)-f_{i}\left(n\right)r\left(n+1\right)\right],\\ y\left(n\right)=\overset{L_{b}}{\underset{i=0}{\prod }}\left|g_{i}\left(n+1\right)v\left(n-1\right)\right|. \end{array}$$

Among them, *L*_*f*_ is the length of the tap coefficients of the feedforward filter, and *L*_*b*_ is the length of the tap coefficients of the feedback filter. The input signal of the equalizer control module includes the input signal of the decider and the output signal of the decider.

### 3.3. Evolutionary Game Adaptive Weighted Fusion Method

Based on the constructed evolutionary game multisource data fusion model, the adaptive weighted fusion of redundant data between homogeneous sensors can be regarded as a noncooperative game process. The self-adaptive weight between each node reflects the competitive relationship between them, and the adjustment process of the weight is the dynamic adjustment process of the fusion game from the nonequilibrium state to the equilibrium state.

In the face of a certain fusion game situation, keeping the strategies of other subjects unchanged, the process that subject *i* achieves utility maximization by changing its own strategy is called the optimal reflection of subject *i* in this game situation. That is, node *i* only generates a new weight distribution by changing its own trust degree, so as to obtain the maximum utility in the current situation. This can actually be regarded as a univariate optimization problem, and we use a simple random mutation process to obtain the optimal response strategy.

The dynamic process in which we let each game subject determine its own optimal response in sequence according to the node number is an optimal response dynamic of game fusion. In the process of adjusting the weights of the adaptive weighted fusion game, the whole system undergoes several rounds of optimal response dynamics, each game subject always constitutes a fixed strategy combination, and the strategy combination constitutes a certain stable state. To avoid getting only a local optimum, we perturb this stable state in a random way to make it regress to the unstable state again.

### 3.4. Acceleration Signal and Its Feature Extraction Method

Through acceleration, the speed and trajectory of human motion can be obtained. In kinematics, when an object is subjected to an external force and a certain displacement occurs in the direction of the force, it is called work. The magnitude of the work can reflect the amount of exercise of the human body, but the physiological impact and fatigue caused by the work should also be considered. If the same task is completed at the same time and with same intensity, the fatigue feeling and physiological performance will be roughly the same each time. In mechanics, the force product can be used to describe the physiological effect of exercise on people.

In this experiment, the tester's handling times were 100 times, and the sampling frequency of acceleration was 50 Hz. In order to facilitate feature extraction and analysis of a large amount of data, the collected and recorded data needed to be divided. The main wave peak of the acceleration signal can reflect the number of times of bending over. Next, the main wave peak of the acceleration signal is extracted to complete the division of the data segment.  Figure 3 shows the feature point extraction of the acceleration signal. Combined with the data characteristics of this experiment, this study compares the adjacent peak points, that is, the peak value is greater than the peak value of its adjacent left and right, and the point is considered as the main peak point.

## 4. Results and Analysis

### 4.1. Numerical Result of Steps

By observing and comparing the experimental data, it is found that the correlation coefficient of these application software for step measurement is relatively high, and the correlation coefficient is 0.991–0.999. The average absolute error percentage of all application software measurement results is relatively small, the average absolute error percentage is 0.23%. −1.98%, and it can be said that the accuracy of the step count measurement value is high and can be used for the step count measurement. Among the five apps, the three apps on the smartphone, Gudong, Dongdong, and LeDong, measure the same number of steps. In the same movement mode, the numerical results obtained by the two bracelets are different, and the numerical results obtained by the mobile phone application software are also different.  Figure 4 shows the comparison of the error rates of the five applications in monitoring normal running steps.

The correlation coefficients of these three software in normal running, fast walking, jogging, and fast running are 0.996, 0.997, 0.991, and 0.997, respectively, and the average absolute error percentages are 1.34%, 1.41%, 1.14%, and 1.98%. When jogging, the correlation coefficients of the five applications were lower compared with other sports, but the average absolute error percentage of the five applications was the smallest when jogging compared with other sports. In running, the correlation and mean absolute error percentage of the two running styles were not significantly different, and the mean absolute error percentage of fast running was higher than that of jogging.

According to the average absolute error percentage, it can be known that the accuracy of the four sports modes is Huawei Band > Xiaomi Band > three mobile phone sports software. At the same time, the results obtained in this experiment are in good agreement with other research results. Observing the steps of the last two subjects, it is found that the average absolute error percentage also meets the requirements of Huawei Band > Xiaomi Band > three mobile phone exercise software, but the average absolute error percentage of this 4,000 meter exercise is smaller than that of the 800 meter exercise. From this, it can be speculated that among the five sports software, the monitoring results of step count in long-distance exercise may be more accurate than in short-distance exercise.

Through observation, it can be found that the average absolute error percentage of Xiaomi Mi Band and Huawei Band is lower than that of the three mobile phone sports software in step monitoring, which may be related to their monitoring principles. The wristband has a built-in acceleration sensor, which can more accurately sense the number of steps, and it can be seen that when the speed increases, that is, the body more accurately swings, but the total number of steps is less than the actual number of steps. This may be due to the inability to record the number of steps when the swing is not significant.

### 4.2. Numerical Results of Movement Distance

The comparison of the error rate of normal running distance monitored by five applications is shown in Figure 5. As the distance of exercise increases, energy expenditure also increases. Therefore, the statistical research of exercise distance is of great significance to the research of energy consumption, especially in the mobile GPS sports software, and the distance statistics are particularly important. Through experimental research, it is known that the distance measurement of these applications is in kilometers and finally accurate to 10 meters, so if you study distance data in short-distance sports, it will inevitably be a bit stretched. All movements in this experiment are fixed at a distance of 800 meters so that the distance can be well compared and analyzed. Since these distance data are fixed values, no correlation analysis can be performed, so the mean absolute error percentage is analyzed in this study.

In the observation of the data of two subjects at 4,000 meters, it is found that the average absolute error percentage is smaller than that at 800 meters, and the accuracy is improved, especially for the three mobile phone sports software. Since the mobile phone sports software is GPS positioning, the distance is more accurate than the bracelet.

### 4.3. Energy Consumption Results of Different Exercise Methods

Figure 6 shows the comparison of the error rates of the five applications for monitoring normal running energy consumption. In normal running, the average absolute error percentages from small to large are Huawei Band, Xiaomi Band, Gudong, Dongdong software, and Le Power. In the fast running exercise, the average absolute error percentages from small to large are Xiaomi Mi Band, Huawei Band, Gudong, Le Power, and Dongdong software. By observing and analyzing the data results, it can be known that among the four sports, the average absolute error percentages of these five software are relatively low during jogging, and the average absolute error percentages of all software for monitoring energy consumption are greater than 1.5%. The error is small in terms of number and distance.

At the same time, the data of the last two 4,000 meter exercise subjects were analyzed, and it was found that the change trend of the average absolute error percentage was the same as the abovementioned normal running results, but the error percentage was reduced. The values monitored by these application software may be more accurate and can be used as a reference for exercisers.

It is worth noting that in the four sports modes, the average value of Codoong and Huawei Band is higher than the average value of the reference value, and the average value of Xiaomi Mi Band is lower than the average value of the reference value. The accuracy of the energy consumption evaluation of different algorithms is shown in Figure 7.

The average absolute error percentages of the five applications in the normal running are all low and less than 25%, the average absolute error percentages of the five applications during fast walking are all low and less than 20%, and the average absolute error percentages of the five applications during jogging are all low. The average absolute error percentages of the five applications are all lower than 35% during brisk walking; the difference between the five application software is not large when jogging; and the difference between the five application software is large during fast running. The mean absolute percent error in all four sports was less than 15%. The energy consumption evaluation time of different algorithms is shown in Figure 8.

### 4.4. Relationship between the Correlation Coefficient between the Application Software and the Actual Energy Consumption Value in Different Stages

Table 1 shows the correlation coefficient between the energy consumption measured by each equipment in normal running. Among them, the correlation coefficient between Gudong and Dongdong software in normal running is 0.99, *P* < 0.01, which is statistically significant; in fast running, the correlation coefficient between Gudong and Huawei Band is 0.863, *P* < 0.01, which has statistical significance. In terms of academic significance, the correlation coefficient between Xiaomi Band and Huawei Band is 0.742, *P* < 0.05, which is statistically significant. The correlation coefficient between the two is 0.762, *P* < 0.05, which is statistically significant; the correlation coefficient between Codoong and Dongdong software in the fast running is 0.888, *P* < 0.01, which is statistically significant. The correlation coefficient was 0.782, *P* < 0.05, which was statistically significant.

## 5. Conclusions

Aiming at the shortcomings of the traditional CMA algorithm, the improved algorithm is studied in detail. In order to solve the error propagation phenomenon of the decision feedback equalizer, an adaptive weighting factor is introduced into the algorithm. In order to solve the shortcomings of the traditional CMA algorithm, a variable-step CMA algorithm based on MSE is also introduced, and finally, an algorithm with better performance is formed. The relationship between the acceleration signal and the amount of human motion is expounded, the original acceleration signal is preprocessed, and then, the time-domain extraction and frequency-domain extraction methods commonly used in acceleration signal analysis are introduced. The significant difference test of the parameters proves the validity of the selected feature parameters. The monitoring of steps by mobile phone exercise software and smart bracelet is highly correlated, which may be related to their principles. The monitoring of steps by smart bracelet and smartphone exercise software is obtained by the internal acceleration sensor of the bracelet and mobile phone. The acceleration changes generated by the internal chip are integrated to output the number of steps, but the relatively small error may be caused by the fact that the body swing is not too small and the arm swing is too small, so that the smartphone and smart bracelet cannot accurately collect information. The distance monitoring error of the mobile phone exercise software is lower than that of the smart bracelet. This study may be due to the fact that the test site is circular, and the final distance may not be detected at the turn, resulting in a low measurement value. When measuring distance and average speed, the smartphone motion software is within 3% of the error of professional equipment, which means that the smartphone motion software has certain advantages in monitoring energy consumption, and the acceleration sensor in the smart bracelet is also very effective in monitoring energy consumption. But these five applications are not very effective in monitoring energy consumption. This may be due to the different calculation methods of energy consumption between smart bracelets and smartphone software, and may also be related to some redundant actions during exercise.

## Figures and Tables

**Figure 1:** CMA-DFE structure diagram.

**Figure 2:** Block diagram of the decision feedback equalizer based on MSE variable step size.

**Figure 3:** Extraction of acceleration feature points.

**Figure 4:** Comparison of the error rates of five applications for monitoring normal running steps.

**Figure 5:** Comparison of the error rate of normal running distance monitored by five application software.

**Figure 6:** Comparison of the error rates of five applications for monitoring normal running energy consumption.

**Figure 7:** Accuracy of energy consumption evaluation of different algorithms.

**Figure 8:** Time-consuming energy consumption evaluation of different algorithms.

**Table 1:** Correlation coefficients between energy consumption measured by various equipment in normal running.

Gudong	Mobile software	Le Power	Xiaomi Bracelet	Huawei Bracelet
Gudong	0.99	0.6	0.62	0.4
Mobile software	—	0.57	0.7	0.6
Le Power	—	—	0.8	0.9
Xiaomi Bracelet	—	—	—	0.7

## Data Availability

The data used to support the findings of this study are available from the corresponding author upon request.
